# Clinical Effect of Abdominal Massage Therapy on Blood Glucose and Intestinal Microbiota in Patients with Type 2 Diabetes

**DOI:** 10.1155/2022/2286598

**Published:** 2022-08-03

**Authors:** Ying Xie, Meng-Ting Huan, Jia-Jia Sang, Song-Song Luo, Xin-Tian Kong, Zhou-Yu Xie, Shi-Hui Zheng, Qing-Bo Wei, Yun-Chuan Wu

**Affiliations:** ^1^College of Acupuncture and Massage, Nanjing University of Chinese Medicine, Nanjing, Jiangsu, China; ^2^Provincial Hospital of Traditional Chinese Medicine, Nanjing, Jiangsu, China; ^3^Changzhou Hospital of Traditional Chinese Medicine, Changzhou, Jiangsu, China

## Abstract

The aim of the study was to investigate the clinical effects of abdominal massage on patients with type 2 diabetes mellitus (T2DM) and its influence on the intestinal microflora. We conducted a randomized, controlled clinical trial. A total of 60 patients with T2DM, who met the inclusion criteria, were randomly allocated to the control group, the routine massage group, and the abdominal massage group. The control group received health education and maintained their hypoglycemic drug treatment plan. The routine massage group and the abdominal massage group received different massage interventions. In addition to glucose and lipid metabolism indicators, we quantitatively analyzed the gut microbiota to assess the effects of massage on the intestinal microflora of patients with T2DM. Compared with the control group, the abdominal massage improved levels of glycated hemoglobin, total cholesterol, Enterobacter, and Bifidobacteria with significant differences (*P* = 0.02, *P* = 0.03, *P* = 0.03, and *P* = 0.03). The comparison within group showed that the levels of the four bacterial genera in the abdominal massage group revealed significant differences before and after treatment (*P* = 0.006, *P* < 0.001, *P* < 0.001, and *P* = 0.002). The comparison between the routine massage group and the abdominal massage group was not significantly different in all levels of test indices. The abdominal massage group regulated levels of Enterobacter and Lactobacilli to a greater extent than the routine massage group. Additionally, abdominal massage decreased Enterococcus levels. The results of this study showed that abdominal massage has clinical advantages over routine massage. Specifically, this intervention may correct microflora disturbances to a certain extent.

## 1. Introduction

Type 2 diabetes mellitus (T2DM) is a chronic metabolic endocrine disease characterized by insulin resistance and insufficient insulin secretion. As a global public health concern, approximately 537 million adults had DM in 2021. The prevalence of DM in obese people continues to increase [1]. However, once patients are diagnosed with T2DM, they can only be treated with long-term maintenance hypoglycemic drugs. In view of the side effects of hypoglycemic drugs, massage therapy, which is safe, effective, and less toxic with few or no side effects, represents a valuable treatment option [2].

Conventional massage consists of regular and rhythmic movements of the therapist's hands on body tissues, including nerves and muscles, to achieve certain goals. Several studies [3–5] have shown that massage improves glucose and lipid metabolism disorders by regulating muscle, inflammatory factors, and pancreatic islet function. Compared with routine massage, abdominal massage is not only easy to perform, but can also improve gastrointestinal function and lipid metabolism [6–9].

Intestinal microflora disorders and abnormal glucose and lipid metabolism are important etiological factors in T2DM [10]. Recent studies show that inflammatory markers are correlated with the diabetic control indices, i.e., glycated hemoglobin (HbA1c) levels in the diabetic population [11]. Not only DM but also its complications such as diabetic nephropathy, frailty, and proteinuria are associated with inflammation [12–14]. On the other hand, the intestinal microbiota has a close relationship with inflammation [15]. Once the intestinal microbiota is imbalanced, it will generate systemic inflammation, which is the characteristic of DM and its complications.

Abdominal massage affects gastrointestinal responses by stimulating parasympathetic nerves [16], but its effectiveness and specific mechanism in the treatment of DM are not clear. It is possible that abdominal massage may modulate the composition of the gut microbiome, thereby affecting metabolism. The objective of this study was to assess the safety and therapeutic effects of abdominal massage in T2DM patients through clinical observation and its effects on the intestinal microflora. Our study findings will provide a basis for understanding the mechanism of abdominal massage in metabolic diseases and the relationship between skeletal muscle movement and the intestinal microflora.

## 2. Materials and Methods

### 2.1. Design

We performed the randomized clinical study following the principles of the Declaration of Helsinki. The study took place between September 2020 and February 2022 after registering it in the Chinese Clinical Trial Registry and obtaining approval from the Ethics Committee of the affiliated hospital of Nanjing University of Traditional Chinese Medicine (2019-210-KY). The trial registration number was ChiCTR2000031688. The subjects were informed about the objectives of the study and provided signed informed consent.

### 2.2. Participants

We recruited 60 patients with T2DM from the massage department of the affiliated hospital of Nanjing University of Traditional Chinese Medicine and the outpatient department of Nanjing Jiqingmen Hospital. We randomly allocated the patients to one of three groups (a control group, a routine massage group, or an abdominal massage group) in a 1 : 1 : 1 ratio. Four patients were lost to follow-up, and two patients were excluded from the study. Therefore, a total of 54 subjects completed the eight-week treatment and follow-up. There were no significant differences in age, course of disease, gender, body weight, or BMI among the three groups (*P* > 0.05; Table 1). Due to the particularity of using conventional hypoglycemic drugs in the control group, it was impossible to blind the subjects and therapists. However, throughout the trial, the data managers, analysts, and evaluators remained blinded to groups to minimize possible confusion of the trial results.

#### 2.2.1. Inclusion Criteria

Patients with all of the following conditions were included in the study: those who meet the diagnostic criteria for patients with T2DM based on the World Health Organization (WHO) diagnostic criteria, the patient is between 35 to 80 years of age, those who agree to the interventions and provide signed informed consent, the patient had not received massage therapy for T2DM during the last 2 weeks, the patient did not participate in other ongoing clinical studies, and the drug regimen for T2DM is metformin alone. Medication for other underlying diseases that are not excluded from the exclusion criteria, assessed by the attending physician and in the patient's own opinion, is acceptable without change during the 2-month trial.

#### 2.2.2. Exclusion Criteria

Patients with one of the following conditions were excluded from the study: type 1 diabetes, late-onset autoimmune diabetes in adults, gestational diabetes, and other secondary diabetes; diseases affecting the cardiovascular, nervous, digestive, or hematopoietic system; or severe metabolic and organic complications of diabetes, such as ketoacidosis and diabetic nephropathy. Additionally, pregnant or lactating women, patients with alcohol or psychotropic substance abuse, and patients with mental illness were excluded. Similarly, patients who had modified the amount and type of drugs consumed within two months before the trial, those who had participated in other clinical trials in the previous two years, those who had consumed antibiotics or micro-ecological drinks within one month before the trial, and those with a weight change of >5% in the first two months of the trial were excluded.

#### 2.2.3. Dropout and Elimination Criteria

The following patients were eliminated from the study: patients who violated the research protocol, who were lost to follow-up, who had additional circumstances that affected the judgment of curative effect, or patients who had poor compliance or withdrew from the study.

### 2.3. Interventions

#### 2.3.1. Control Group

Patients were provided with health education, guidance on healthy eating habits, and exercise. The routine hypoglycemic drug treatment plan was maintained. The intervention continued for eight weeks.

#### 2.3.2. Routine Massage Group

The treatment was based on “Tuina Therapeutics” by Professor Fan Binghua [17]. Firstly, the patient was in a prone position, and the therapist performed chiropractic sessions five times. The therapist pressed and kneaded the bladder meridian, focusing on BL13, BL20, BL21, BL22, and BL23 for three minutes each. Subsequently, they rubbed BL23 and BL31-34 to diathermy, pinched and pushed from both lower limbs to the Achilles tendon three times, and pressed and rubbed KI1 to diathermy. Secondly, the patient was in a supine position. A one-finger Zen push method was applied to the Ren meridian, focusing on RN15, RN13, RN12, RN6, and RN4. This session was performed three times. The holding method from the front of both lower limbs to the ankle joints was performed twice. The therapist tapped GB34, ST36, and SP6 for one minute each. Lastly, the patient was in a seated position. The therapist kneaded GB20, DU16, and DU20 by thumb for one minute each. Subsequently, they pinched the neck and GB21 for one minute each and tapped the shoulder and back once. The whole procedure lasted approximately 30 minutes, three times a week, one time every other day, for eight weeks, with rest on Sundays.

### 2.4. Abdominal Massage Group

The selection and manipulation of acupoints in the abdominal massage group were derived from clinical experience. First, the patient laid on their back. The therapist pressed and rubbed RN13, RN12, and RN10 for five minutes each. Second, at 30 r/min, the therapist rubbed the abdomen in a clockwise manner for 15 minutes. Third, the therapist used the one-way holding method from ST21 to ST29 on both sides. Four, the therapist rubbed under the flank to induce diathermy. The whole procedure lasted approximately 30 minutes, three times a week, once every other day, for eight weeks, with rest on Sundays.

### 2.5. Test Indices

The patients fasted after 21 : 00 in the evening. We collected venous blood on an empty stomach at 7 : 00 the next morning once before and after treatment. Fasting blood glucose (FPG) and postprandial blood glucose (PBG) were measured using the glucose oxidase method. High performance liquid chromatography was used to detect glycated hemoglobin (HbA1c). Total cholesterol (TG), triglycerides (TG), high-density lipoprotein (HDL), and low-density lipoprotein (LDL) were measured using an automatic biochemical analyzer (HITACHI 3100, China). Fluorescence quantitative PCR was used to detect Enterococcus, Enterobacter, Bifidobacterium, and Lactobacillus. Before and after treatment, fresh fecal specimens from the middle and back sections of all test patients were collected in the morning and quickly stored at −80 °C. DNA extraction was completed within 24 h after sampling. The sample library construction, sequencing, and analysis services were completed by China Shanghai Meiji Pharmaceutical Biotechnology Co, Ltd.

### 2.6. Statistical Analysis

We performed statistical analysis using SPSS22.0 software. The Shapiro-Wilk test was used in the normality analysis of the study. We expressed normally distributed data with homogeneity of variance as mean ± standard deviation (SD). Using the Chi-square test, we analyzed the count data. When the measurement data met the requirements of normal distribution and homogeneity of variance, the paired *t*-test was used for the comparison of the two samples within the group before and after treatment, the independent *t*-test was used for the comparison between the groups, one-way analysis of variance was used for comparison of multiple groups, and the LSD method was used for pairwise comparison between groups. A rank-sum test was used for those who did not meet the requirements, and a nonparametric test was used for comparison of multiple groups of sample data. We set statistical significance at *P* < 0.05.

## 3. Results

We randomly allocated 60 patients with T2DM to one of three groups: control, routine massage, or abdominal massage group. Four patients dropped out, and two patients were excluded from the study. Therefore, a total of 54 patients completed the trial. The number of cases in the control, routine massage, and abdominal massage groups was 17, 18, and 19, respectively. The dropout and elimination rates from the three groups were analyzed using the Chi-square test. The rates of dropout and elimination were comparable (*P* = 0.57; Table 2).

### 3.1. Baseline Characteristics

There were no differences in age (*P* = 0.87), disease duration (*P* = 0.67), gender (*P* = 0.87), body weight (*P* = 0.40), and BMI (*P* = 0.33) among the three groups (Table 1).

### 3.2. Data Analysis of Efficacy Indicators before and after Treatment

#### 3.2.1. Comparison of FBG, PBG, and HbAlc Indexes

When comparing before and after treatment within a group, we observed that the levels of FBG, PBG, and HbAlc had no statistical differences in the control group and were significantly different in the abdominal massage and routine massage groups (control: *P* = 0.07, *P* = 0.09, and *P* = 0.31; abdominal massage: *P* < 0.001, *P* < 0.001, and *P* < 0.001; and routine massage: *P* < 0.001, *P* < 0.001, and *P* < 0.001). Pairwise comparison between groups showed that there were significant differences between the control group and the abdominal massage group in the level of HbAlc (*P* = 0.02) and there were no significant differences between the control group and the routine massage group and between the routine massage group and the abdominal massage group in the levels of FBG, PBG, and HbAlc (*P* = 0.14, *P* = 0.19, *P* = 0.11; *P* = 0.68, *P* = 0.97, and *P* = 0.40) (Table 3).

FBG, PBG, and HbAlc values in the routine massage and abdominal massage groups were lower after the intervention. The clinical efficacy of the abdominal massage in reducing the level of HbAlc was higher than no massage (control).

#### 3.2.2. Comparison of TC and TG Indexes

When comparing before and after treatment within a group, we observed that the level of TC had no statistical difference in the routine massage group and was significantly different in the control and abdominal massage groups (*P* = 0.07, *P* = 0.01, and *P* = 0.005). The level of TG had no statistical differences in all groups (control: *P* = 0.27; abdominal massage: *P* = 0.27; and routine massage: *P* = 0.60). Pairwise comparison between groups showed that, when compared with the control group, the abdominal massage and routine massage groups were significantly different in the level of TC (*P* = 0.03 and *P* = 0.046) and had no statistical differences in the level of TG (*P* = 0.83 and *P* = 0.66). Compared with the routine massage group, the abdominal massage group had no statistical difference in the levels of TC and TG (*P* = 0.76 and *P* = 0.52) (Table 4).

Therefore, the level of TC in the control and abdominal massage groups decreased after treatment. The clinical efficacy of the abdominal massage in reducing the level of TC was higher than no massage.

### 3.3. Comparison of HDL and LDL Indexes

When comparing before and after treatment within a group, we observed that the level of HDL had no statistical difference in the abdominal massage and routine massage groups and was significantly different in the control group (*P* = 0.43, *P* = 0.20, and *P* = 0.002). The level of LDL was significantly different in all groups after treatment (control: *P* = 0.01; routine massage: *P* = 0.049; and abdominal massage: *P* = 0.02). Pairwise comparison between groups showed that, when compared with the control group, the abdominal massage group was significantly different in the levels of HDL (*P* = 0.046) and the abdominal massage and routine massage groups had no statistical differences in their levels of LDL (P = 0.10, P =0.11). Compared with the routine massage group, the abdominal massage group had no statistical difference in the levels of HDL and LDL (*P* = 0.39 and *P* = 0.90) (Table 5).

Therefore, the level of LDL in all groups decreased after treatment, and the level of HDL decreased only after no massage treatment. The clinical efficacy of the abdominal massage in reducing the level of LDL had no difference with routine massage and control groups.

### 3.4. Observation Index Data Analysis before and after Treatment

#### 3.4.1. Comparison of Enterococcus and Enterobacter Indexes

When comparing before and after treatment within a group, we observed that the level of Enterococcus had no statistical differences in the control and routine massage groups (*P* = 0.65 and *P* = 0.38), and the level of Enterobacter had no statistical difference in the control group and was significantly different in the routine group (*P* = 0.93 and *P* = 0.03). The levels of both bacteria were significantly different in the abdominal massage group (P =0.006, P <0.001). Pairwise comparison between groups showed that, when compared with the control group, the abdominal massage and routine massage groups had no statistical differences in their levels of Enterococcus (*P* = 0.32 and *P* = 0.75). The abdominal massage group was significantly different, and the routine massage group had no statistical difference in the level of Enterobacter (*P* = 0.03 and *P* = 0.41). Compared with the routine massage group, the abdominal massage group had no statistical difference in the levels of both bacteria (*P* = 0.50 and *P* = 0.17) (Table 6).

Therefore, the level of Enterobacter in the routine massage and abdominal massage groups decreased after treatment, and the level of Enterococcus decreased only after abdominal massage treatment. The clinical efficacy of the abdominal massage in reducing the level of Enterobacter was higher than no massage.

#### 3.4.2. Comparison of Bifidobacteria and Lactobacilli Indexes

When comparing before and after treatment within a group, we observed that the levels of Bifidobacteria and Lactobacilli had no statistical difference in the control group and were significantly different in the routine massage and abdominal massage groups (control: *P* = 0.23 and *P* = 0.56; routine massage: *P* < 0.001 and *P* = 0.04; and abdominal massage: *P* < 0.001 and *P* = 0.002). Pairwise comparison between groups showed that, when compared with the control group, the abdominal massage group was significantly different and the routine massage group had no statistical difference in the level of Bifidobacteria (*P* = 0.03 and *P* = 0.06). The abdominal massage and routine massage groups had no statistical differences in their levels of Lactobacilli (*P* = 0.59 and *P* = 0.66). Compared with the routine massage group, the abdominal massage group had no statistical difference in the levels of both bacteria (*P* = 0.82 and *P* = 0.31) (Table 7).

Therefore, the levels of Bifidobacteria and Lactobacilli in the abdominal massage and routine massage groups increased after treatment. The clinical efficacy of the abdominal massage in reducing the level of Bifidobacteria was higher than no massage.

## 4. Discussion

T2DM presently has no known treatment. Injections of insulin plus the usage of oral hypoglycemic medications make up the standard treatment for diabetes mellitus (DM). The drawbacks and side effects of these treatments, however, include gastrointestinal issues, anemia, liver and kidney damage, and lactic acid toxicity [18].

Massage is one of the most popular and effective methods for relaxation and therapy [19]. Manual massage is commonly used in the treatment of pathological conditions affecting the skeletal muscles [20–22]. Recently, mechanisms by which massage is beneficial for the musculoskeletal system have been investigated. According to the findings, massage has an immunomodulatory effect on skeletal muscles, affecting protein and ribosome synthesis and degradation, anabolic signaling, and satellite cell abundance [23]. The effects of manual massage have been classified as reflexive, mechanical, and psychological, resulting in vasodilation and improved circulation [24]. Interestingly, massage induces skin microcirculation, expands blood vessels and improves blood flow, promotes insulin secretion, improves the nervous system and the function of the vegetative nervous system, enhances the immune function and metabolism of the body, and promotes the utilization of glucose by muscle tissue, thereby reducing blood sugar levels [25, 26]. As a complementary treatment strategy, it is crucial to explore the most effective massage method in the treatment of T2DM.

Abdominal massage, also named visceral massage in China, involves mechanical and manual manipulations that are used in the treatment of prediabetes, overweight, and obesity [27]. Numerous studies have shown that abdominal massage reduces thigh, infraumbilical, arm, and post-partum abdominal circumference; decreases flank subcutaneous fat deposits and serum lipid lipids; and improves skin laxity [28–30]. Additionally, the effects on gastrointestinal function have been extensively studied [31]. The function of abdominal massage in lipid metabolism and gastrointestinal function suggests that it could be beneficial in the treatment of T2DM.

Our study findings revealed that both abdominal and routine massage reduce the levels of FBG, PBG, and HbAlc. Besides, abdominal massage improves the levels of TC and LDL. It proved the regulative effects of massage on glucose and lipid metabolism disorders in patients with T2DM. In addition, these interventions can increase the number of beneficial bacteria (e.g., Bifidobacteria and Lactobacillus) and reduce the number of pathogenic bacteria (e.g., Enterococcus and Enterobacter). Dysbiosis is a causative factor in T2DM because it affects energy metabolism and storage and promotes chronic inflammation. In terms of energy [32], the intestinal microflora improves glucose and lipid metabolism by producing short-chain fatty acids, encouraging fat synthesis and storage, and so on. In contrast, intestinal dysbiosis generates the production of endotoxins, leading to systemic inflammation, destruction and apoptosis of pancreatic *β* cells, and insulin resistance [33]. In this study, abdominal massage modulated the intestinal microbiota in T2DM patients, although more research is required to determine the precise mechanisms. We measured three laboratory indices to determine the impact of abdominal massage on glucose metabolism (FBG, PBG, and HbAlc). Future research should evaluate the pancreatic islet function and insulin resistance indexes.

The ability to regulate intestinal microflora suggests that there are interactions between the skeletal muscle and the gut microbiota during abdominal massage. Manual abdominal massage includes different techniques directed to the abdominal soft tissues, including kneading, friction, rubbing, and pinching. This intervention involves the passive movement of abdominal skeletal muscles and of the rectus abdominis, internal oblique, external oblique, and transverse abdominis. According to the evidence, muscular disorders may arise from microbial factors that trigger innate immunity and low-grade systemic inflammation [34]. On the other hand, the metabolic and inflammatory states, muscle function, and gut microbiota are all interconnected [35]. Active skeletal muscle exercise, such as that used in fitness, has been shown to affect the composition and activity of the microbiota in studies using human and animal models [36, 37]. We verify that improving the gut microbiota's equilibrium can be accomplished by passive abdominal skeletal muscle activity. Thus, abdominal massage therapy is a complementary form of treatment for T2DM.

## 5. Conclusion

In patients with T2DM, abdominal massage significantly reduced abnormalities in the intestinal microbiota and glucose metabolism. Abdominal massage was simpler to do than regular massage because it did not require changing the patient's body posture. Abdominal massage is quite convenient for both doctors and patients, especially given the increased prevalence of DM in obese persons. This study will advocate abdominal massage as a trustworthy treatment option for T2DM patients.

## Figures and Tables

**Table 1:** Characteristics of participants (*χ* ± s).

Group	Number (male/female)	Age (y)	Duration (y)	Weight (kg)	BMI (kg/m^2^)
Control	17 (7/10)	64.24 ± 9.24	6.88 ± 6.26	66.91 ± 8.82	25.66 ± 1.12
Routine massage	18 (9/9)	67.50 ± 6.72	8.11 ± 7.88	67.57 ± 6.93	25.20 ± 1.25
Abdominal massage	19 (9/10)	63.11 ± 6.83	6.16 ± 5.59	70.27 ± 7.81	26.00 ± 2.18
*P* value	0.87	0.21	0.67	0.40	0.33

**Table 2:** Number of dropouts or eliminated participants.

Group	Number	Dropouts or eliminated	*P* value
Control	17 (85.0%)	3 (15.0%)	
Routine massage	18 (90.0%)	2 (10.0%)	0.57
Abdominal massage	19 (95.0%)	1 (5.0%)	

**Table 3:** Comparison of FBG, PBG, and HbAlc values before and after treatment (*χ* ± s).

Groups	FBG (mmol/L)		PBG (mmol/L)		HbAlc (%)	
	Before	After	Before	After	Before	After
Control	8.02 ± 0.96	7.70 ± 0.88	11.28 ± 1.82	10.59 ± 1.86	7.20 ± 0.59	7.13 ± 0.60
Routine massage	8.63 ± 1.44	7.21 ± 1.08^∗∗^	13.02 ± 2.60	9.74 ± 1.86^∗∗^	7.53 ± 0.98	6.68 ± 0.83^∗∗^
Abdominal massage	8.76 ± 1.63	7.08 ± 0.92^∗∗^	13.19 ± 3.16	9.72 ± 1.96^∗∗^	7.49 ± 1.17	6.45 ± 0.97^∗∗#^
*F* value	1.40	2.03	2.88	1.21	0.63	3.13
*P* value	0.26	0.14	0.07	0.31	0.54	0.05

Comparison within group, ^∗^*P* < 0.05 and ^∗∗^*P* < 0.01. Comparison with control group, ^#^*P* < 0.05 and ^##^*P* < 0.01.

**Table 4:** TC and TG levels before and after treatment (*χ* ± s).

Group	TC (mmol/L)		TG (mmol/L)	
	Before	After	Before	After
Control	4.43 ± 1.09	3.86 ± 0.71^∗^	2.12 ± 2.72	1.68 ± 1.64
Routine massage	5.01 ± 0.93	4.50 ± 0.70^#^	2.13 ± 1.04	1.93 ± 1.02
Abdominal massage	5.52 ± 0.65	4.59 ± 0.61^∗∗#^	2.24 ± 2.44	1.55 ± 1.00
*F* value	3.37	3.36	0.01	0.22
*P* value	0.05	0.05	0.99	0.80

Comparison within group, ^∗^*P* < 0.05 and ^∗∗^*P* < 0.01. Comparison with control group, ^#^*P* < 0.05 and ^##^*P* < 0.01.

**Table 5:** HDL and LDL levels before and after treatment (*χ* ± s).

Group	HDL (mmol/L)		LDL (mmol/L)	
	Before	After	Before	After
Control	1.19 ± 0.26	1.04 ± 0.22^∗∗^	2.73 ± 0.84	2.23 ± 0.50^∗^
Routine massage	1.21 ± 0.10	1.18 ± 0.12	3.03 ± 0.81	2.59 ± 0.47^∗^
Abdominal massage	1.31 ± 0.34	1.27 ± 0.35^#^	3.24 ± 0.55	2.62 ± 0.52^∗^
*F* value	0.59	2.22	1.08	1.92
*P* value	0.56	0.13	0.35	0.17

Comparison within group, ^∗^*P* < 0.05 and ^∗∗^*P* < 0.01. Comparison with control group, ^#^*P* < 0.05 and ^##^*P* < 0.01.

**Table 6:** Enterococcus and Enterobacter levels before and after treatment (*χ* ± s).

Group	Enterococcus (LogN/g)		Enterobacter (LogN/g)	
	Before	After	Before	After
Control	8.53 ± 0.85	8.48 ± 0.56	9.38 ± 0.67	9.38 ± 0.61
Routine massage	8.48 ± 0.98	8.39 ± 0.78	9.34 ± 1.07	9.16 ± 0.89^∗^
Abdominal massage	8.53 ± 1.10	8.22 ± 0.97^∗∗^	9.19 ± 0.85	8.81 ± 0.74^∗∗#^
*F* value	0.01	0.53	0.24	2.56
*P* value	0.99	0.59	0.79	0.09

Comparison within group, ^∗^*P* < 0.05 and ^∗∗^*P* < 0.01. Comparison with control group, ^#^*P* < 0.05 and ^##^*P* < 0.01.

**Table 7:** Bifidobacterium and Lactobacillus levels before and after treatment (*χ* ± s).

Group	Bifidobacteria (Log N/g)		Lactobacilli (Log N/g)	
	Before	After	Before	After
Control	8.13 ± 0.59	8.05 ± 0.58	6.84 ± 0.91	6.79 ± 0.92
Routine massage	8.10 ± 0.73	8.51 ± 0.77^∗∗^	6.32 ± 1.19	6.63 ± 1.16^∗^
Abdominal massage	8.07 ± 0.65	8.56 ± 0.74^∗∗#^	6.64 ± 1.29	6.99 ± 1.09^∗∗^
*F* value	0.04	2.84	0.91	0.52
*P* value	0.96	0.07	0.41	0.60

Comparison within group, ^∗^*P* < 0.05 and ^∗∗^*P* < 0.01. Comparison with control group, ^#^*P* < 0.05 and ^##^*P* < 0.01.

## Data Availability

The study data are available upon request. We welcome specific proposals for future collaboration.
